The article "Accurate 3D Reconstruction of White Matter Hyperintensities Based on Attention-Unet" was published in 2022. Journal: Comput Math Methods Med.

# Accurate 3D Reconstruction of White Matter Hyperintensities Based on Attention-Unet

**DOI:** 10.1155/2022/3812509

**Published:** 2022-03-23

**Authors:** Xun Wang, Lisheng Wang, Jianjun Yang, Xiaoya Feng

**Affiliations:** ^1^College of Computer Science and Technology, China University of Petroleum (East China), Qingdao, 266580 Shandong, China; ^2^Department of General Practice, Shandong Provincial Third Hospital, Shandong University, Jinan, 250031 Shandong, China; ^3^Department of Neurology, Shandong Provincial Third Hospital, Shandong University, Jinan, 250031 Shandong, China

## Abstract

White matter hyperintensities (WMH), also known as white matter osteoporosis, have been clinically proven to be associated with cognitive decline, the risk of cerebral infarction, and dementia. The existing computer automatic measurement technology for the segmentation of patients' WMH does not have a good visualization and quantitative analysis. In this work, the author proposed a new WMH quantitative analysis and 3D reconstruction method for 3D reconstruction of high signal in white matter. At first, the author using ResUnet achieves the high signal segmentation of white matter and adds the attention mechanism into ResUnet to achieve more accurate segmentation. Afterwards, this paper used surface rendering to reconstruct the accurate segmentation results in 3D. Data experiments are conducted on the dataset collected from Shandong Province Third Hospital. After training, the Attention-Unet proposed in this paper is superior to other segmentation models in the segmentation of high signal in white matter and Dice coefficient and MPA reached 92.52% and 92.43%, respectively, thus achieving accurate 3D reconstruction and providing a new idea for quantitative analysis and 3D reconstruction of WMH.

## 1. Introduction

The decline of cognitive function, the risk of cerebral infarction, and dementia seriously affect the health of modern people. At present, there are many methods to predict cognitive decline and cerebral infarction dementia. Qiao and others believe that MMSE prediction plays an important role in the early detection of Alzheimer's disease. They use the convolutional neural network to predict MMSE more effectively [1]. Solovyev and others believe that the decline of cognitive ability is related to Alzheimer's disease and capillary stagnation and the convolutional neural network should be used to detect capillaries, which achieves good results [2]. In recent years, the quantitative analysis of white matter hyperintensity (WMH) has attracted extensive attention. White matter hyperintensities (WMH), also known as white matter osteoporosis, are characterized by high signal in T2-weighted magnetic resonance imaging (MRI) FLAIR or T1W sequence images and fluid attenuation inversion recovery sequences. The pathological changes are mainly noncharacteristic white matter injury, manifested as membrane discontinuity, glial cell proliferation, white matter fiber looseness, pale or swelling of myelin sheath, diffuse axonal injury, and vacuole formation [3, 4]. It was confirmed by the clinic that WMH is associated with cognitive decline, risk of cerebral infarction, and dementia and with gait disorders, balance disorders, and urinary incontinence. Except that, studies have shown that more than 90% of people over the age of 60 have white matter hyperintensities.

The existing WMH quantitative analysis methods at home and abroad are semiautomatic measurement, and doctors need to supervise the whole process. In addition, the existing methods cannot directly display the reconstruction effect and cannot well assist doctors in quantitative analysis. Hernández et al. [5] proposed and evaluated the indicators of white matter damage and realized the quantitative assessment of WMH. Muhammad et al. [6] proposed a convolutional neural network to segment conventional WMH and achieved good results. Dadar et al. [7] used the machine learning method to achieve the segmentation of WMH and reached the Dice coefficient of 0.84. However, the existing computer automatic measurement technology for the segmentation of patients' WMH does not have a good visualization and quantitative analysis and the reconstruction has not yet retrieved relevant reports.

Medical imaging equipment, such as CT and MRI, can obtain two-dimensional digital tomography images of internal organs of the human body but cannot display the three-dimensional structure of objects. The 3D reconstruction technology in computer image processing and graphics can reconstruct the 2D medical image sequence in 3D and can simulate and display the 3D structure of organs. The human body is scanned by medical scanning imaging equipment, and a continuous two-dimensional digital picture of the fault is obtained, which is then fed into a computer and read. Feature enhancement and segmentation were performed on the fault sequence images. After that, the segmented region is used to reconstruct the 3D image using the reconstruction algorithm. How to conduct accurate segmentation and 3D reconstruction of WMH is a problem that needs to be solved in this paper.

WMH accurate segmentation is the first step in 3D reconstruction. At present, most of the segmentation methods targeting the lesions are still in their infancy. Clustering method is one of the most commonly used traditional segmentation methods. It mainly realizes pixel clustering through the feature similarity of the pixels in the target region. In addition, traditional methods such as the Bayesian classifier and support vector machine (SVM) are also commonly used in lesion segmentation. However, the traditional methods of lesion segmentation usually have the characteristics of complex training and poor segmentation accuracy. With the development of deep learning technology, it is often used in medical image segmentation and detection and has achieved ideal results. In 2015, Long et al. [8] used the convolutional layer to extract features and used the deconvolutional layer to decode the feature image and restore it to the size of the input image, thus realizing image per-pixel classification. After the introduction of FCN, a series of convolutional network structures have been designed for image pixel classification, such as SegNet [9], DeepLabv3 [10], and Unet [11]. These networks are structurally composed of two parts, the coding layer and the decoding layer, and the structure is clear and easy to understand. Among them, Unet has been widely used in the segmentation of medical lesions [12–16] and achieved good results. Extraction of lesion features is the basis of accurate segmentation. VGG-16 [17] and GoogleNet [18] are commonly used lesion feature extraction networks, but their redundant network layer learns parameters that are not identity mapping, resulting in network degradation, while ResNet [19] solves the above model degradation problem by designing residual modules and achieve better feature extraction.

The current 3D reconstruction methods are generally divided into two kinds: surface rendering and volume rendering. In this paper, 3D reconstruction of segmented WMH is performed based on surface rendering. In the early stage of medical scanning imaging equipment, the distance between sections is relatively large and the slice-level surface reconstruction is generally adopted. With the improvement of medical scanning and imaging equipment technology, surface reconstruction based on voxel appears. The isosurfaces are extracted by some algorithms, and the isosurfaces are drawn by constructing the geometric elements of the isosurfaces in the voxels. Yu [20] used 3D reconstruction technology to reconstruct traumatic atlantoaxial vertebra, so as to better help doctors specify appropriate surgical methods. He [21] reconstructed continuous heart tissue sections and realized virtual heart visualization.

In this paper, the improved Unet is used to segment the WMH and the ResNet structure is added on the basis of WMH. In addition, the attention mechanism of CBAM [22] was added in this paper to achieve feature extraction of WMH. In order to solve the ambiguity problem caused by 3D reconstruction with the moving cube method, we used the moving tetrahedron method for 3D reconstruction of a series of segmented images. In this paper, the author conducted data experiments on 23742 pathological images of 100 patients in Shandong Province Third Hospital. The location of the lesion was marked by a professional radiologist. According to the radiologist's labeling, 702 CT images with high white matter signal were selected. The data experiments show that the segmentation network proposed in this paper, compared with other popular segmentation networks, has at least 0.01 Dice coefficient improvement, which also provides the basis for accurate 3D reconstruction of WMH. In addition, the effect of 3D reconstruction in this paper is greatly improved compared with other methods. Through literature analysis, this is the first attempt to carry out accurate 3D reconstruction of WMH and provides a new idea for quantitative analysis and reconstruction of WMH.

## 2. Materials and Methods

### 2.1. Materials

The dataset in this paper was obtained from Shandong Province Third Hospital, China, including 100 patients with a total of 23742 pathological images. The locations of lesions were marked by professional radiologists. In this paper, 702 CT images with white matter hyperintensities were selected according to the radiologist's annotation. Due to the high contrast between WMH and surrounding tissues, FLAIR sequences have higher clarity and integrity compared with T1W and T2W sequences. In this paper, most of the DICOM images of high signal in white matter were selected from FLAIR sequence and a few were selected from other sequences.

In the experiment, the white matter hyperintensity data is divided into the train set and test set according to the ratio of 8 : 2. The train set is used for the training of white matter hyperintensity image segmentation, and the test set is used for segmentation test.

The accuracy of white matter hyperintensity reconstruction depends on the accuracy of segmentation. In this paper, the author use histogram equalization to enhance white matter hyperintensity data. The segmentation accuracy of high signal in white matter was greatly improved.

### 2.2. Methods

#### 2.2.1. Model

The series of the Unet network is a kind of image segmentation network based on the convolutional neural network. Compared with the traditional full convolutional neural network, Unet has been improved to achieve full extraction of features through stronger connection between layers, plus upsampling and downconvolution. To better focus on dividing the area, ResUnet adds jump connection on the basis of Unet to better improve the accuracy of the deep convolutional neural network.

As shown in Figure 1, ResUnet is a U-shaped symmetrical structure, with the convolution layer on the left and the upper sampling layer on the right. Same as Unet, ResUnet contains 4 convolution layers and the corresponding 4 upper sampling layers and the feature map obtained from each convolution layer will be connected to the corresponding upper sampling layer, so that the feature map of each layer can be effectively used in the subsequent calculation. The corresponding upper sampling layer and convolution layer are calculated with a convolution kernel of 3 × 3 size and activated with ReLu. Among them, 4 convolution layers are connected by a 2 × 2 maximum pool and 4 upper sampling layers are upsampled by 2 × 2 convolution kernel. In addition, ResNet adds jump connections in each convolution layer and upper sampling layer, which are shown in Figure 1 as solid blue arrows. ResUnet with jump connection has better segmentation effect, which has been verified in the experiment. In addition, this paper adds a CBAM attention module after each convolution layer and upper sampling layer, so that the network can obtain better segmentation effect. CBAM is covered in more detail in the next section. The white matter hyperintensity CT images enter the ResUnet network, pass through multiple convolution layers and upper sampling layers, and finally get the accurate segmentation results.

ResUnet uses the Dice loss function to achieve pixel-level segmentation of high signal in white matter. Dice coefficient is derived from dichotomy and is essentially a measure of the overlap of two samples. The Dice function is shown as follows:

(1) $$\begin{array}{c} \text{Dice}=\frac{2\;|\;A\cap B\;|\;}{\;|\;A\;|\;+\;|\;B\;|\;}. \end{array}$$

Among them, ∣*A*∩*B*∣ represents the common elements between set *A* and set *B*, ∣*A*∣ represents the number of elements in the set *A*, and ∣*B*∣ denotes the number of elements in set *B*. In this paper, the original target and the segmented target are overlapped at pixel level to obtain their Dice value.

#### 2.2.2. CBAM Attention Mechanism

According to the experimental results of Yu [20], sequential addition of channel attention and spatial attention was carried out in this paper. For channel attention, feature graphs generated at the last layer will be maximized and average pored, to generate different spatial context descriptors *F*_max_^*c*^ and *F*_avg_^*c*^. The descriptor is then entered into the shared network MLP, and the resulting eigenvectors are merged by a summation operation.

The formula for channel attention is as follows:

(2) $$\begin{array}{c} C\left(F\right)=\begin{array}{c} \sigma \left(\text{MLP}\left(\text{AvgPool}\left(F\right)+\text{MLP}\left(\text{MaxPool}\left(F\right.\right.\right)\right)\\ \sigma \left(W_{1}\left(W\left(F_{\text{avg}}^{c}\right)\right)+W_{1}\left(W_{0}\left(F_{\max}^{c}\right)\right)\right) \end{array}, \end{array}$$

in which *σ* represents sigmoid function, *W*_0_ and *W*_1_ are weights in the MLP-shared network, where *W*_0_ ∈ ℝ^*C*/*r*×*C*^ and *W*_1_ ∈ ℝ^*C*×*C*/*r*^, and *r* represents the reduction rate, aiming at reducing parameter calculation in the shared network.

For spatial attention, the formula is as follows:

(3) $$\begin{array}{c} S\left(F\right)=\sigma \left(f^{7\times 7}\left(\left[\text{AvgPool}\left(F\right);\text{MaxPool}\left(F\right)\right]\right)\right),\\ =\sigma \left(f^{7\times 7}\left(\left[F_{\text{avg}}^{s};F_{\max}^{s}\right]\right)\right), \end{array}$$

in which *σ* represents sigmoid function and *f*^7×7^ represents convolution operation with a filter size of 7 × 7.

#### 2.2.3. WMH Reconstruction

After accurate segmentation of white matter hyperintensities, the segmentation images of each group were reconstructed in 3D.

The Marching cubes algorithm is a classic algorithm among surface rendering algorithms. It is a voxel level reconstruction algorithm proposed by Lorense [23] in 1987, also known as the isosurface extraction algorithm. The main idea of the moving cube algorithm is to approximate the isosurface by linear difference in a three-dimensional discrete data field. In medical image segmentation and reconstruction, this isosurface is determined by defining a threshold value. First, define the concept of a “cell,” as distinct from a “voxel.” A voxel is a grid of eight pixels arranged in sequence, and each voxel (except the boundary) is shared by the eight voxels. There are three kinds of vertex values in a volume element: above or equal to the value is inside the surface, and below the value is outside the surface. Move the cube as shown in Figure 2.

As shown in Figure 2, *l*_*k*_ and *l*_*k*+1_ represent two different isosurfaces; (*i*, *j*, *k*) represent the vertices of voxels. There are two possible states for one vertex of a voxel, so a voxel (8 vertices) has a total of 28 or 256 states, where the grayscale value of a point within the voxel (as in Figure 2) can be calculated using the trilinear interpolation equation (4).

(4) $$\begin{array}{c} f\left(x,y,z\right)=a_{0}+a_{1}x+a_{2}y+a_{3}z+a_{4}xy+a_{5}yz+a_{6}zx++a_{7}xyz. \end{array}$$

*a*_0_ − *a*_7_ represent the gray value of the eight vertices of the voxel; *x*, *y*, *z* represents the coordinate points in the voxel; *f* (*x*, *y*, *z*) represents the gray value of the points (*x*, *y*, *z*) in the voxel. The 256 combinations can be reduced to 128 combinations by reversing the symmetry (the exchange of vertex 0 and 1 values in the boundary voxel). By rotating the symmetry (the position of vertexes 0 and 1 is the same after the rotation of the boundary voxel), the 256 combinations can be reduced to 15 cases. Each state of the volume element contains a number of three facets, and the vertices of the triangular facets in the volume element need to be calculated by linear interpolation according to the value of the isosurface and the value of the two vertices on the side.

In order to solve the problem of ambiguity in the connection of triangular surfaces in the moving stereoscopic method, this paper uses the moving tetrahedron method [24, 25] to carry out 3D reconstruction. Compared with the moving stereo method, the moving tetrahedron algorithm is to divide the cube element in the moving cube algorithm into tetrahedrons. There are many ways of splitting, usually dividing into 5 tetrahedrons, and then constructing isosurfaces in the tetrahedron. There are 24 and 16 combinations in total. By inverting and rotating symmetry, only one vertex in the boundary voxel is larger than the isosurface, so the triangular surface is generated. If two vertices are larger than the isosurface, a quadrilateral surface is generated, as shown in Figure 3.

Figure 3 shows the schematic diagram of the moving tetrahedron method. The article uses the moving tetrahedron method for 3D reconstruction of the white matter of the brain and is able to achieve better modeling accuracy.

## 3. Results

### 3.1. Evaluation Metrics

In this paper, segmentation and 3D reconstruction were performed on the white matter hyperintensity (WMH) dataset. In order to assess the accuracy of 3D reconstruction relative to the gold standard manual label, a number of corresponding measures for various volumes and spaces were used in this article, as no single measure reflects all the required information about the quality of the reconstruction. In this paper, Dice coefficient is mainly used as the evaluation index of spatial correspondence of each voxel between two segments. Dice coefficient can measure the similarity between WMH output from the segmented network and real samples. Among them, the Dice coefficient value is between 0 and 1 and the larger the value is, the closer the segmentation is to the real value. The Dice coefficient formula is as follows:

(5) $$\begin{array}{c} \text{Dice}\left(S,Y\right)=\frac{2\;|\;S\cap Y\;|\;}{\;|\;S\;|\;+\;|\;Y\;|\;}. \end{array}$$

Among them, the prediction result of the segmentation network is ∣*S*∣ and the real result is ∣*Y*∣. The intersection of the two results is represented by ∣*S*∩*Y*∣. In addition, in order to evaluate the accuracy of segmented pixels, MPA (average pixel accuracy) is also used to analyze the experimental results of the two types of pixels in the process of WMH segmentation. The MPA value is also between 0 and 1. The higher the value, the higher the pixel accuracy. MPA formula is as follows:

(6) $$\begin{array}{c} \text{MPA}=\frac{1}{n_{cl}}\overset{n_{cl}}{\underset{i=0}{\sum }}\frac{P_{ii}}{\sum_{j=0}^{n_{cl}}P_{ij}}. \end{array}$$

The number of categories is expressed in *n*_*cl*_, the number of correctly classified pixels is expressed in *p*_*ii*_, and the pixels with wrong classification are expressed in *p*_*ij*_. In this paper, different models are used for experimental comparison to prove the effectiveness of the module added in this paper for WMH segmentation. All models are trained on the obtained WMH training set and evaluated on the verification set.

### 3.2. Implementation Details Jinan Science and Technology Bureau

For the sake of equality and comparison, all the real tests are carried out on PyTorch codes. The actual training was conducted on a Ubuntu 16.04 operating system with 6x Intel(R) Core (TM) i7-7700 CPU, and a NVIDIA GeForce RTX 2080 GPU was used for training. The image input size of each network is 512 × 512 pixels. In addition, this paper sets 30 epoch for the training of each network model and sets the initial learning rate of each model to 0.001. Unless otherwise stated, all models use the same parameters.

### 3.3. Main Results

In this paper, MPA and Dice coefficients are used as the evaluation indexes of the spatial correspondence of each voxel between the two segmentations. Due to the lack of WMH data, this paper uses TTA (test time augmentation) to enhance the results of the test set and uses the way of fivefold cross-validation. By observing the results obtained by using the method in this paper, the effect of corresponding WMH reconstruction is evaluated. In addition, in order to prove the effectiveness of the improvement of the Unet model in this paper, an experimental comparison was conducted on SegNet, DeepLabv3, and Unet.

The experimental results are shown in Table 1.

SegNet achieves a MPA of 86.34% and a Dice coefficient of 87.43% in the segmentation of white matter hyperintensity intensity. Similarly, DeepLabv3 has a MPA of 90.65% and a Dice coefficient of 91.31%, which is higher than SegNet, while the Attention-Unet used in this paper has a Dice coefficient of 92.52%, which is higher than other flow line segmentation models. In addition, compared with Unet, the residual module and CBAM attention module added in this paper increase the Dice coefficient by 2.15% and 1.47%, respectively. This is enough to prove the accuracy of the segmentation method used in this paper.

In order to better represent the content of the experimental results, the segmentation effects of five different models are compared and the comparison effect is shown in Figure 4.

Among them, WMH segmentation and reconstruction effects obtained by Attention-Unet and the moving tetrahedron method are shown in Figure 5, where WMH is generated from the segmented images of this sequence.

## 4. Discussion

In this paper, an accurate 3D reconstruction of WMH is attempted for the first time and a new idea for quantitative analysis and reconstruction of WMH is provided. In order to make the results of 3D reconstruction more accurate, this paper proposes an attention-based model called Attention-Unet. The model adds attention mechanism to achieve more accurate white matter hyperintensity segmentation and improve the accuracy of 3D reconstruction. The experimental results show that the Dice coefficient and MPA of the model on WMH dataset are 92.52% and 92.43%, respectively, which is better than the current popular segmentation model, thus laying an important foundation for the realization of accurate 3D reconstruction. In the following work, the author will try to achieve accurate measurement of the volume of 3D reconstruction of white matter hyperintensities, so that it can be applied to clinical work more quickly. In the next work, we will refer to the following novel work [26–32] to try to improve the accuracy of 3D reconstruction of the WMH and the speed of segmentation.

## Figures and Tables

**Figure 1:** The model of Attention-Unet.

**Figure 2:** Schematic diagram of moving the cube.

**Figure 3:** Schematic diagram of the quadrilateral surface.

**Figure 4:** WMH segmentation effects of different models.

**Figure 5:** Segmentation and reconstruction renderings. (a, b) Are the results of segmentation of a group of WMH images. (c) Represents the 3D reconstruction result obtained from the segmented image.

**Table 1:** Results of each model experiment (mean ± s.d.%).

Method	Reference module		Evaluation coefficient	
	ResNet	CBAM	Dice (%)	MPA (%)
SegNet	✘	✘	87.43 ± 0.92	86.34 ± 0.58
DeepLabv3	✘	✘	91.31 ± 0.67	90.65 ± 1.08
Unet	✘	✘	88.90 ± 0.43	86.26 ± 1.12
ResUnet	✔	✘	91.05 ± 0.37	90.81 ± 0.49
Attention-Unet	✔	✔	92.52 ± 0.16	92.43 ± 0.82

## Data Availability

The data supporting the study are available in the database https://github.com/wls860707495/-White-Matter-Hyperintensities
